RETRACTED

# Long Noncoding RNA LINC00857 Promotes Proliferation, Migration, and Invasion of Colorectal Cancer Cell through miR-1306/Vimentin Axis

**DOI:** 10.1155/2021/5525763

**Published:** 2021-03-23

**Authors:** Na Chang, Yayun Cui, Xue Liang, Dan Han, Xiaomin Zheng, Ailin Wu, Liting Qian

**Affiliations:** Department of Radiation Oncology, Anhui Provincial Cancer Hospital (West District, The First Affiliated Hospital of USTC, Division of Life Sciences and Medicine, University of Science and Technology of China), Hefei, Anhui 230031, China

## Abstract

Colorectal cancer is a commonly diagnosed cancer and the leading cause of cancer-related death which still increasing in many countries. The lack of biomarkers for early detection and clinic treatment results in high morbidity and mortality. The novel role of long noncoding RNA LINC00857 on cell proliferation migration and invasion was explored in this article. The expression level of LINC00857 in colorectal cancer tissue samples and cells was determined notably higher than normal tissue samples and cells. Silence LINC00857 can significantly inhibit colorectal cancer cell viability and metastasis in vitro. Moreover, LINC00857 depletion caused cell accumulation in the G0/G1 phase. In addition, we recognized the novel LINC00857–miR-1306–vimentin axis and demonstrated it by dual-luciferase reporter assay. And this signaling axis could be considered as the target for colorectal cancer treatment. In conclusion, LINC00857 can promote colorectal cancer progress by sponging miR-1306 and upregulate vimentin to accelerate the epithelial-mesenchymal transition process.

## 1. Introduction

Presently, more than 945,000 people develop colorectal cancer which is a kind of malignant tumor and cause more than 492,000 patients to die every year in worldwide [1]. According to researches, up to 20% of colorectal cancer patients existed metastasis disease, which usually occurs in the liver [2]. The most common therapeutic strategies for colorectal cancer are surgical resection and chemotherapy. And this is not an effective treatment for colorectal cancer obviously [3]. Recently, advances in the molecular subtypes, methylation of DNA, and microRNA biogenesis in colorectal cancer result in the identification of many new biomarkers in colorectal cancer diagnosis [4]. And many novel strategies like immunotherapy have also shown a promising prospect for colorectal cancer treatment [5]. Therefore, the recognition and application of new biomarkers in early detection and clinic treatment would improve the prognosis for colorectal cancer patients.

As a kind of noncoding RNA, lncRNA has been demonstrated involved in many biological reactions in cells, especially in cancer cells [6]. Upregulated or downregulated lncRNA can promote or inhibit cell proliferation, apoptosis, migration, and invasion as well as cancer cell stemness by regulating gene expression at epigenetic, transcriptional, and posttranscriptional level [7]. In recent years, the function of many long noncoding RNA has been explored in many cancer types. LINC01793 was demonstrated upregulated in gastric cancer and probably act as the key molecule to promote gastric cancer development [8]. lncRNA FOXD2-AS1 was also detected in various cancers, like lung, gastric, colorectal, bladder, thyroid, hepatocellular, skin cancer, and esophageal. The result indicated lncRNA FOXD2-AS1 was overexpressed in these cancers and accelerate tumor progress [9]. Therefore, exploration of the function and the underlying mechanism of these lncRNAs in various cancers would help us to recognize the target for early prognosis and treatment.

RETRACTED

Linc00857, as a long noncoding RNA, has been determined upregulated in many cancer types and can promote tumor progression. In hepatocellular carcinoma, LINC00857 can accelerate tumor development. Silencing LINC00857 in hepatocellular carcinoma cells will significantly decrease the viability and block the cell cycle in G1 phase [10]. In muscle-invasive bladder cancer, high expression of LINC00857 was correlated with shorter recurrence-free and poor overall survival of patients [11]. In lung cancer, knockdown of LINC00857 will notably suppress tumor progression through inhibiting cancer cell growth, migration, and invasion [12]. However, there is no related research focused on this lncRNA in colorectal cancer so far.

Recently, more and more evidence has revealed the role of mRNA-miRNA-lncRNA networks in a variety of human cancers. lncRNA is usually the precursor RNA of microRNA (miRNA) or acts as a competitive endogenous RNA (ceRNA) to interact with miRNA [13]. In breast cancer, lncRNA HOTAIR affects the growth, metastasis, and apoptosis of breast cancer cells through the miR-20a-5p/HMGA2 axis [14]. lncRNA-RMRP can promote the proliferation, migration, and invasion of bladder cancer cell lines by regulating miR-206 as a sponge, becoming a potential target for the treatment of bladder cancer patients [15]. In non-small-cell lung cancer (NSCLC), lncRNA-ATB promotes the apoptosis of NSCLC cells by inhibiting the expression of miR-200a and promoting the expression of *β*-catenin [16].

Therefore, we designed experiments to explore the function and mechanism of LINC00857 in colorectal cancer. Firstly, we collected colorectal cancer tissue samples and cells to detect the expression level of LINC00857 compared with normal tissues and cells. Secondly, we performed CCK-8 assay, transwell assay, and cytometry cell cycle assay to determine whether LINC00857 can decrease the cell viability and metastasis in colorectal cancer cells. Lastly, we recognized the down-stream microRNA and the target gene by dual-luciferase reporter assay. The result explained why LINC00857 can promote cancer cell metastasis and why LINC00857 is a crucial role in tumor development.

RETRACTED

## 2. Materials and Methods

### 2.1. Sample and Cell Line Collection

18 cases of colorectal cancer patients admitted to Anhui Provincial Cancer Hospital were involved in this study. All patients expressed their full intent to participate, and their written informed consent was obtained. The procedure was approved by the Medical Ethics Committee of the Anhui Provincial Cancer Hospital. Human colorectal cancer cell lines (RKO and HCT-116) and the normal colorectal epithelial cell line FHC were procured from ATCC (Manassas, VA, USA). The cells were cultured in RPMI-1640 (BI, Israel) supplied with 10% fetal bovine serum (FBS, Gibco) in a humidified incubator containing 5% CO_2_ at 37°C. All cell lines were shown negatively in mycoplasma experiment and regularly authenticated by short tandem repeat profiling. Collect cells at 90% confluence and change the medium every 48-72 hours.

### 2.2. Cell Transfection

The siRNA which targets LINC00857 was procured from Genepharma Co. (Shanghai, China). For transfection, cells (1 × 10^5^ per well) were seeded into six-well plates and infected by lipofectmine2000 (Invitrogen, Thermo, USA) for 6 hours before use. Si-LINC00857/NC, miR-1306/NC mimics, and vimentin/empty vector plasmid use Lipofectamine 2000 (Invitrogen, Carlsbad, California) according to the manufacturer's instructions. After infection, the cell was harvested, and the transfection efficacy was determined by qRT-PCR.

### 2.3. RNA Extraction and Quantitative Real-Time PCR

Total RNA of the colorectal cancer specimens and cell lines was extracted by using the Trizol method (TaKaRa, Dalian, China). RNA was reverse transcribed by using PrimeScript RT Master Mix (Perfect Real Time) (TaKaRa) and then amplified using the SYBR Green PCR Kit (Vazyme, Nanjing, China). GAPDH and U6 genes are used as endogenous control genes to normalize the expression of target genes. Each sample was analyzed in triplicate. The expression levels of target genes were measured using 2^-*ΔΔ*CT^ method.

### 2.4. Cell Proliferation Detection

Cell counting kit 8 (CCK-8, Dojindo Chemical Laboratory, Kumamoto, Japan) was used to detect the proliferative capacity of colorectal cancer cells. Cells (2 × 10^3^ per well) were seeded in 96-well plates, and the cell viability was determined according to the CCK-8 manufacturer's instructions.

RETRACTED

### 2.5. Transwell Assay

The migration and invasion capacities of colorectal cancer cell lines were detected using Transwell chambers (Corning, NY, USA) either with Matrigel (for invasion assays) or without Matrigel (for migration assays). Cells (3 × 10^4^) were plated to upper insert in 100 *μ*L of serum-free RPMI-1640, and 600 *μ*L of RPMI-1640 medium containing 10% FBS was added into the lower chamber. After 24 hours, cells remaining on the upper chamber were removed with cotton swabs and that had adhered to the lower surface of the membrane were fixed with methanol and stained with DAPI for 10 min. Then, the invaded and migrated cell lines were photographed and counted under light microscopy.

### 2.6. Cell Cycle Analysis

For cell cycle analysis, G1, S, and G2 peaks were detected from the propidium iodide-stained GC cells by flow cytometry (Beckman, Brea, CA, USA), and the Modfit software was used for analysis.

### 2.7. Dual-Luciferase Reporter Assay

The wild-type and mutant sequences of LINC00857 or 3′UTR of vimentin were inserted into luciferase vector (Promega, Madison, Wisconsin) and cotransfected with Renilla luciferase using Lipofectamine 2000 (Invitrogen, Carlsbad, California). After 48 hours of transfection, the luciferase activities were determined with the Dual-Luciferase Reporter Assay System (Promega, Madison, Wisconsin) according to the manufacturer's instructions.

### 2.8. Statistical Analysis

All experiments were repeated three times. The SPSS 20.0 software was used to analyze all representative data. All the derived data was indicated as mean ± SD. Differences that existed in two comparison groups or multiple groups were calculated by Student's *t*-test. *P* value less than 0.05 indicated a significant difference.

## 3. Results

### 3.1. lncRNA LINC00857 Is Overexpressed in Colorectal Cancer Cell Lines and Tissues

At first, we detected the expression of LINC00857 in colorectal cancers. In this study, 18 colorectal cancer tissues were subjected for detection. The clinical colorectal cancer tissues from 18 patients indicated notably higher LINC00857 expression compared with the adjacent normal tissues (Figure 1(a)). FHC, a normal colorectal epithelial cell line, was used in this study. After that, we determined the relative expression level of LINC00857 in different colorectal cancer cells.  Figure 1(b) indicates that LINC00857 expression level in the HCT-116 and RKO cells was significantly increased compared with that in the FHC cell. These data reveal that LINC00857 is significantly overexpressed in human colorectal cancers.

### 3.2. SiRNA Infection Is Highly Efficient against LINC00857

We design and synthesize siLINC00857 to knock down LINC00857 in HCT-116 and RKO cells. Then, colorectal cancer cells were transfected with siLINC00857 targeted LINC00857 or siNC as a negative control.  Figure 1(c) indicates high transfection efficiency in the RKO and HCT-116 cells. Next, we determined the expression level of LINC00857 in RKO and HCT-116 cells. The level of LINC00857 was decreased by 87% in the RKO cells infected with siLINC00857 compared to the siNC-transfected cells. In HCT-116 cell, the LINC00857 expression level was descended to 23% of the negative control. These data indicate the high efficiency of the siRNA to knock down the LINC00857 expression in cells.

RETRACTED

### 3.3. LINC00857 Knockdown Decreases Cell Viability In Vitro

Firstly, we performed cell fractional was conducted by using PARIS™ Kit (AM1921, Invitrogen, USA). And real-time PCR was applied to detect the expression level of LINC00857 in nucleus and cytoplasm. The result showed LINC00857 was mostly located in cytoplasm (Figures 2(a) and 2(b)). We determined the function of LINC00857 in colorectal cancers. The CCK-8 assay revealed there is no significant difference in the first and second days for RKO and HCT-116 cells. However, the proliferation rate was significant suppressed in HCT-116 cells which transfected with siLINC00857 on the third day, and the difference continued to increase in the next 2 days in HCT-116 cells (Figure 2(c)). The significant difference in proliferation rate also appeared in the fourth and fifth days in the RKO group (Figure 2(d)). These data demonstrate that LINC00857 can promote colorectal cancer cell proliferation in vitro.

### 3.4. LINC00857 Knockdown Results in Cell Cycle Inhibition in Colorectal Cancer Cells

To examine the impact of LINC00857 knockdown on cell cycle in RKO and HCT-116 cells, flow cytometry cell cycle analysis was conducted. After incubating for 24 h, the cells were collected and then stained with PI. The result was monitored and analyzed by flow cytometry. In RKO cell, LINC00857 knockdown promotes cells increased in the G0/G1 phase but decreased in the S phase (Figure 3(a)). Similarly, with transfected with siLINC00857, HCT-116 cells which stay in the S phase shifted to the G0/G1 phase significantly (Figure 3(b)). This result shows that knockdown of LINC00857 arrested cell cycle in the G0/G1 phase in both the RKO and HCT-116 cells.

### 3.5. LINC00857 Facilitates Colorectal Cell Migration and Invasion *In Vitro*

We detected the effect of LINC00857 knockdown on cancer cell metastasis by performing migration and invasion assays. In this assay, many RKO and HCT-116 cells were migrated to the surface of the low chamber, with a significant disparity between cells which transfected with siNC or siLINC00857 (Figure 4). These data demonstrate that LINC00857 can facilitate cell metastasis in vitro.

RETRACTED

### 3.6. miR-1306 Can Directly Bind with LINC00857 and Target the EMT-Associated Protein Vimentin

We used miRcode (http://www.mircode.org/) and TargetScan 7.1 database (http://www.targetscan.org) to predict the binding sites between LINC00857 and miR-1306 and the target genes of miR-1306. To determine whether LINC00857 can directly bind with miR-1306, we constructed luciferase reporter plasmid. The miR-1306 mimic and the reporter plasmid contain LINC00857 wild-type or mutant were transfected into 293T cell line. The data suggest the luciferase activity of LINC00857 wild-type reporter was notably inhibited by miR-1306 mimic (Figure 5(a)). However, the luciferase activity of LINC00857 mutant reporter does not have a significant difference with miR-1306 mimic (Figure 5(a)). Besides, vimentin luciferase reporter or vimentin mutant reporter plasmid was cotransfected into 293T cells with miR-1306 mimic. Data suggest miR-1306 can also directly bind with vimentin in cell (Figure 5(b)).

EMT was demonstrated to play an important role in colorectal tumorigenesis and development. During this process, mesenchymal marker vimentin often increases its expression, whereas epithelial marker E-cadherin loses its overexpression [17]. In this experiment, we demonstrated that LINC00857 could sponge and suppress miR-1306 which can directly target vimentin. Due to the upregulation of LINC00857 in colorectal cancer, the expression level of vimentin was also increased, and therefore, colorectal cancer cell metastasis was promoted.

### 3.7. Rescue Vimentin in Colorectal Cancer Cells Could Reverse Inhibitory Effect of Proliferation by LINC00857 Knockdown and miR-1306 Overexpression

Vimentin expression level was positively correlated with LINC00857 and inhibited by miR-1306 in colorectal cancer cell was demonstrated before. In rescue assay, we overexpressed vimentin in colorectal cancer cells which was transfected siLINC00857 or miR-1306 mimics. Quantitative real-time PCR determined expression level of vimentin was significantly recovered compared with only knockdown LINC00857 or overexpress miR-1306 group (Figures 5(c) and 5(d)). By performing CCK-8 assay, results shown knockdown LINC00857 or overexpress miR-1306 notably reduced viability in colorectal cancer cells, and overexpress vimentin would reverse this result (Figures 5(e)–5(h)). Totally, overexpress vimentin in colorectal cancer cells would significantly reverse the suppressive effect by LINC00857 knockdown or miR-1306 overexpression in viability. These results suggest that LINC00857-miR-1306-vimentin probably was a crucial pathway for LINC00857 to regulate colorectal cancer genesis and progress. And this would be regarded as a novel target for colorectal cancer diagnosis and treatment.

RETRACTED

## 4. Discussion

Presently, colorectal cancer is the third most common cancer which diagnosed in the US [18]. Though the incidence is decreasing in developed countries, there is evidence indicating that the incidence will still notably increase in many developing countries, like China, Croatia, and Costa Rica [19]. EMT, epithelial-mesenchymal transition, a process of cancer cell partially loses the epithelial marker and partially gains the mesenchymal marker to promote cancer cell metastasis [20]. Recently, EMT has emerged as the key regulator to facilitate cancer cell migration and invasion to the distant organs. And this is the most crucial factor of poor prognosis and low overall survival rate of cancer patients [21].

Long noncoding RNA, which was demonstrated, can regulate cancer progress and sponge microRNA in cell [22]. lncRNA XLOC_009167 was demonstrated highly expressed in lung cancer to promote cancer development and was considered as a novel biomarker of lung cancer to be applied in clinical detection [23]. In this article, we collected colorectal cancer tissues and cells to determine the level of LINC00857 by qRT-PCR. The result indicates that LINC00857 is highly expressed in colorectal cancer cells and tissues compared with normal cells and tissues. Then, we performed CCK-8 assay and demonstrated that LINC00857 can significantly increase the viability of colorectal cancer cell in vitro. The flow cytometry analysis showed that cell cycle was blocked by LINC00857 knockdown, and transwell assay indicated that silence LINC00857 can remarkably inhibit cell metastasis in colorectal cancer cell lines. We also recognized that miR-1306 would directly bind with LINC00857 and target vimentin in cell. So we performed dual-luciferase reporter assay, and we demonstrated that LINC00857 can sponge miR-1306 and positively regulate vimentin. These data prove that LINC00857 is a crucial regulator in the development and cancer cell metastasis of colorectal cancer.

Vimentin, an important mesenchymal marker that was demonstrated, overexpressed in many cancer types to accelerate cancer cell migration [24]. And the regulation of vimentin is actually complex due to the posttranslational modifications like phosphorylation and cleavage by intracellular proteases [25]. Based on previous studies, considering vimentin as a target for clinical treatment and a biomarker applied in early prognosis would be practicable [26, 27]. Vimentin has been considered as a marker of EMT [28]. Vimentin functions during cell migration to maintain structure and movement. In gastric cancer (GC), FOXK1 and vimentin have been found to act synergistically to promote GC invasion and metastasis by inducing EMT [29]. Twist1 regulates vimentin to promote EMT in hepatocellular carcinoma [30]. In our research, LINC00857 was proved that can positively regulate vimentin through sponge miR-1306. This could be the reason of why inhibited LINC00857 in colorectal cancer cell can significantly decrease cell migration and invasion. And the LINC00857–miR-1306–vimentin signaling axis could be a novel target to against colorectal cancer.

RETRACTED

This study has a limitation. The expression levels of miR-1306 and vimentin should be detected in clinical samples. In future studies, we will collect more clinical samples and clinical parameters to explore the correlation between miR-1306 and vimentin expression and clinical parameters (including clinical stage, age, and survival rate). In addition, we will further explore the sponge effect of LINC00857 on miR-1306, including RNA pull-down assay and RIP assay, to further clarify the mechanism of LINC00857 in colorectal cancer.

In conclusion, LINC00857 is a novel long noncoding RNA that can promote colorectal cancer cell cycle, cell growth, migration, and invasion. LINC00857 can also sponge miR-1306 and therefore regulate vimentin in cells. Inhibit LINC00857 would be a novel and feasible strategy for colorectal cancer treatment.

## Figures and Tables

**Figure 1:** LINC00857 was determined highly expressed in colorectal cancer tissues and cell lines compared with normal tissues and cell lines. (a) Quantitative real-time PCR was performed to detect the expression level of LINC00857 in colorectal cancer tissues (*n* = 18) and the adjacent normal tissues (*n* = 18). ^∗^*P* < 0.05. (b) LINC00857 expression level in colorectal cancer cell lines (RKO and HCT-116) and normal colorectal epithelial cell line (FHC) was determined by qRT-PCR. ^∗∗∗^*P* < 0.001, ^∗∗∗∗^*P* < 0.0001. (c) SiLINC00857 was used in LINC00857 knockdown in cell, and control group was transfected with siNC. The efficiency of knockdown was detected by qRT-PCR. ^∗∗∗∗^*P* < 0.0001.

**Figure 2:** Silence LINC00857 can inhibit colorectal cancer cell proliferation in vitro. (a, b) The location of LINC00857 was detected by using PARIS kit and quantitative real-time PCR in HCT-116 and RKO cells. U6 was considered as nuclear control, and GAPDH was considered as cytoplasmic control for standardized. (c) Cell count kit-8 was applied to measure the viability of colorectal cancer cells between LINC00857 knockdown and control group in HCT-116 cell. ^∗∗^*P* < 0.01, ^∗∗∗^*P* < 0.001. (d) Cell count kit-8 was applied to measure the viability of colorectal cancer cells between LINC00857 knockdown and control group in RKO cell. ^∗∗^*P* < 0.01.

RETRACTED

**Figure 3:** LINC00857 knockdown result in colorectal cancer cell cycle arrested in G0/G1 phase. (a) Flow cytometry analysis of cell cycle was performed to analyze the cell cycle when LINC00857 was inhibited compared with the control group in RKO cell. ^∗∗^*P* < 0.01, ^∗∗∗^*P* < 0.001. (b) Flow cytometry analysis of cell cycle was performed to analyze the cell cycle when LINC00857 was inhibited compared with control group in HCT-116 cell. ^∗∗∗^*P* < 0.001, ^∗∗∗∗^*P* < 0.0001.

**Figure 4:** Colorectal cancer cell metastasis was decreased with LINC00857 depletion. Invasion and migration assays were performed to detect the colorectal cancer cell metastasis when LINC00857 was depleted compared with the control group. ^∗∗∗∗^*P* < 0.0001.

**Figure 5:** miR-1306 was demonstrated can directly bind with LINC00857 and vimentin in cell. (a) miR-1306 was demonstrated can directly bind with LINC00857 in cell by dual-luciferase reporter assay. ^∗∗^*P* < 0.01. (b) miR-1306 was demonstrated can directly bind with vimentin in cell by dual-luciferase reporter assay. ^∗∗^*P* < 0.01. (c) Vimentin was overexpressed in RKO and HCT-116 cells with LINC00857 knockdown to rescue the expression level of vimentin. ^∗^*P* < 0.05, ^∗∗∗^*P* < 0.001. (d) Vimentin was overexpressed in RKO and HCT-116 cells with miR-1306 overexpressed to rescue the expression level of vimentin. ^∗^*P* < 0.05, ^∗∗^*P* < 0.01. (e–h) Overexpress vimentin in RKO and HCT-116 cells could reverse the inhibitory effect on cell viability from LINC00857 knockdown or miR-1306 overexpression by performing CCK-8 assay. ^∗^*P* < 0.05, ^∗∗^*P* < 0.01.

## Data Availability

The data used to support the findings of this study are available from the corresponding author upon request.

## Abbreviations

EMT: Epithelial mesenchymal transition
qRT-PCR: Quantitative real time polymerase chain reaction
mRNA: Messenger RNA
miRNA: MicroRNA
CCK-8: Cell counting kit 8.
